# The Effect of Nonpharmacological Integrated Care Protocols on Patients with Fatigue Undergoing Hemodialysis: A Randomized Controlled Trial

This article has been retracted.

**DOI:** 10.1155/2022/1047959

**Published:** 2022-10-17

**Authors:** Manhua Zuo, Na Zuo, Jinrong Lin, Jing Zhuo, Xinghui Jing, Jun Tang

**Affiliations:** ^1^Department of Nursing, Zhuhai Campus of Zunyi Medical University, No. 368 Jinwan Road, Sanzao Town, Jinwan District, Zhuhai, Guangdong, China; ^2^Hemodialysis Central, Suining Central Hospital, Suining, Sichuan, China; ^3^Department of Foreign Languages, Zhuhai Campus of Zunyi Medical University, No. 368 Jinwan Road, Sanzao Town, Jinwan District, Zhuhai, China; ^4^Teaching Department of Humanities and Social Science, Zhuhai Campus of Zunyi Medical University, No. 368 Jinwan Road, Jinwan District, Zhuhai, Guangdong Province, China; ^5^Department of Nephrology, The Fifth Affiliated Hospital, Zhuhai Campus of Zunyi Medical University, No. 1439 Zhufeng Avenue, Doumen District, Zhuhai, Guangdong, China

## Abstract

This study was designed to investigate the effects of nonpharmacological integrated care protocols on fatigue in patients with hemodialysis. This parallel randomized controlled trial was conducted on patients undergoing hemodialysis from May to October 2020 at the Dialysis Center of the Fifth Affiliated Hospital of Zunyi Medical University. The patients were randomized into an intervention group (accepting nonpharmacological integrated care protocols and standard care) or a control group (accepting standard care only) using a computer-generated random number. The nonpharmacological holistic care intervention used in this study involved a well-rounded multidisciplinary team that worked together to improve dietary compliance, medication adherence, and self-management to improve patients' care and promote self-management. From the 120 evaluated patients, 116 cases were eligible and analyzed. The results showed that patients from the intervention group had obviously reduced overall fatigue, mental fatigue, and muscular fatigue relative to the control group. The nonpharmacological integrated care protocols were interactive and promotive to each other. Meanwhile, the role and function of nurses in the management of chronic disease were demonstrated to be crucial.

## 1. Introduction

Despite technological advances in the treatment of patients undergoing hemodialysis, they remain subject to major health problems. Fatigue, which often displays as tiredness and lack of energy, is a burdensome symptom with a high estimated prevalence (60-97%) in hemodialysis patients [1]. However, the overall fatigue burden on dialysis days is usually worse than on nondialysis days. Meanwhile, fatigue may create extreme mental and physical debilitation that considerably affects social interaction, quality of life, and well-being [2]. Despite this, the importance of fatigue in hemodialysis patients is still not recognized, and its management remains challenging [3].

Fatigue is usually grouped into two types: muscular and mental fatigue [4, 5]. Mental fatigue can be as serious as muscular fatigue in patients undergoing hemodialysis [6]. Nevertheless, most prior studies on the treatment of fatigue have focused on improving muscular fatigue rather than mental fatigue [7]. In addition, services to address mental fatigue in hemodialysis patients are sporadic because psychological interventions rely on specialized psychological experts, and most dialysis nurses do not have qualifications in psychotherapy. Therefore, integrated intervention protocols, including intervention of nonspecialized qualifications in psychology, were established.

The ability of people to perform normally (physically and mentally) is hindered by fatigue, which is regarded as a subjective and unpleasant symptom that can range from tiredness to exhaustion. Moreover, patient independence and everyday activities are restricted by fatigue, which is also frequently viewed as a cause of stress and linked to a lower quality of life. The treatment-related factors and involved diseases, such as dialysis intensity and frequency, medication, anemia, and inflammation, are frequently blamed for fatigue in patients on dialysis. No drug is discovered to affect or lessen feelings of fatigue, with the exception of injections of erythropoietin to prevent anemia. Research demonstrates that fatigue is not sorely induced by physiological factors, despite the fact that it is usually believed to be a physiological side effect of chronic diseases. Actually, a complex interplay of behavioral manifestations, psychosocial phenomena, and biological processes appears to be the root reason of fatigue. A number of social, psychological, and behavioral factors, like (lack of) social support, depression, stress, anxiety, physical inactivity, substance use, and sleep disorders, are identified by previous research to influence the fatigue in long-term dialysis patients. Another research brought attention to the complicated characteristics of fatigue in patients with end-stage renal disease (ESRD). A distinction among affective, cognitive, and physical fatigue was made by the authors who also listed various dialysis-related, psychological, sociodemographic, behavioral, and physiological factors that may have an impact on those different dimensions of fatigue. Patients on dialysis may experience less fatigue with nonpharmacological interventions that focus on social, cognitive, psychological, and behavioral factors [8].

Our previous research [6] and related literature [9] showed that the physiological, psychological, and social causes were predictors of fatigue in hemodialysis patients, thus considering fatigue as a multifaceted symptom. The National Kidney Foundation (NKF) (2005) and the Kidney Disease Improving Global Outcomes (KDIGO) [10] recommended 30 min of physical activity on most days of the week for patients with renal disease, and the National Academy of Sports Medicine (NASM) characterizes home-based walking as a mild to moderate intensity physical activity. Meanwhile, a low level of cognitive skills in self-management for patients on hemodialysis may lead to poor dietary adherence and other suboptimal self-care, which is associated with compromised health outcomes [11]. However, health education in behavioral self-management is widely used to support management in patients with chronic illnesses including diabetes mellitus by enhancing cognitive self-management skills to develop healthy behavior [12]. On the other hand, motivational interviewing (MI) by individuals without psychotherapist qualifications has been widely conducted to facilitate change in a range of health behavior in patients with chronic diseases [13].

Therefore, this research established nurse-led nonpharmacological integrated care protocols based on physiological, psychological, and social factors to investigate the impact of the protocols in reducing fatigue and improving other indicators in hemodialysis patients.

## 2. Methods

### 2.1. Study Design and Participants

We followed the methods of Dr. Wieke E. van der Borg [8]. A randomized parallel-controlled pilot study was conducted at the dialysis center of the nephrological department in the Affiliated Hospital of University from May to October 2020. The study was carried out following the Declaration of Helsinki. All participants who could withdraw from this study anytime offered the informed consent. The biomedical ethics committee of West China Hospital (2016-23) reviewed and approved this study, with a prospective registration of trial in the Chinese Clinical Trial Registry (ChiCTR-IOR-16008621).

Participants were assigned at random to one of the intervention group (integrated care protocols with standard care) and the control group (standard care only) via a computer-generated randomization list with the ratio of intervention group *vs.* control group being 8 : 7 applied by the researcher who was not involved in the recruitment or outcome collection. The study flow is displayed in Figure 1. Four of the 120 patients who had been screened were later dropped out, leaving 116 patients who ultimately underwent analysis following the 6-month intervention.

### 2.2. Screening Criteria

The inclusion criteria were listed: (1) outpatient hemodialysis patients with good psychological abilities and able to comprehend and communicate; (2) fatigue score ≥ 1 on the Revised Piper Fatigue Scale (RPFS) for patients receiving hemodialysis [14, 15]; (3) aged ≥18 years; (4) had received ≥3 months of hemodialysis and had a stable disease status (unchanged for at least 3 months) and treatment protocols (not changed during 3 months and above for the same patient); (5) patients who walked ≤30 min/day [16]; and (6) could walk independently and free of arthrosis.

The study exclusion criteria were as follows: (1) recently suffered heart or brain vascular diseases such as cardiac insufficiency, myocardial infarction, severe arrhythmia, unstable angina, or stroke; (2) recently had unstable, acute, or critical central or peripheral nervous system diseases, serious infection, or cerebrovascular disease; and (3) blood pressure > 170/110 mmHg as measured with a Riva-Rocci sphygmomanometer in the hospital.

### 2.3. Intervention

The nurse-led nonpharmacological integrated care protocols were based on the rationales of the Theory of Unpleasant Symptoms [17], which integrates the causes of chronic diseases involving three common factors: physiological, psychological, and situational factors. Therefore, the following integrated care protocols were established based on the following. (1) Walking [18, 19]: among patients' daily walking steps were ensured ≥6000 steps, which were counted with a Meilen pedometer. The Meilen pedometer was hung vertically from the belt or the waistband of the trousers except during bathing and sleeping for a six-month period from the beginning to the last day of this study. (2) Health education in behavioral self-management [11] was delivered using spoken language, paper brochures, simulations, and audiovisual presentations in sessions of 45 min each, conducted twice a month. (3) MI [20] was applied in sessions of 20 min each, once monthly per person. The study was conducted for a six-month period. The integrated care protocols were designed and delivered by a multidisciplinary team.

People received standard care with compliance on diet, drinking, and treatments in the control group, while those in the intervention group received the nonpharmacological holistic intervention combined with standard care.

### 2.4. Outcome Measures

Sociodemographic data were collected by research assistants at the beginning of the study, and fatigue, clinical indicators, and other symptom level data were collected at two times points, the beginning and the end of this study.

#### 2.4.1. Primary Outcomes

Due to the high prevalence of fatigue profoundly and negatively impacting the overall health and well-being of patients undergoing hemodialysis, the primary outcome was fatigue, which was assessed using the RPFS, a 22-item and 10-point scale with a range from 0 (indicating no fatigue) to 10 (indicating severe fatigue). Based on the latter scale, total scores had a range of 0 to 10, determined by dividing the total item scores by the total number of items. Scores of 0, 1-3, 4-6, and 7-10 indicated no symptoms, mild symptoms, moderate symptoms, and severe symptoms, respectively. The fatigue symptoms were more severe when the scores were higher. The range of the total Cronbach's alpha on this scale was from 0.80 to 0.99.

#### 2.4.2. Secondary Outcomes

The secondary indicators, obtained from electronic medical records, were the vitality level (evaluated using the SF-36 scale [21]), anxious and depressive level (evaluated using the Hospital Anxiety and Depression Scale (HADS) [22]), sleeping level (evaluated using the Pittsburgh Sleep Quality Index (PSQI) [23]), perceived social support level (evaluated using the Perceived social support scale (PSSS) [24]), and the self-management behavioral level (evaluated using the Behavioral Self-Management Scale [25]). The characteristic of each scale was as follows.

The entire SF-36 scale comprised 36 items and 8 dimensions (subscales). The method of Li et al. was adopted to calculate the total scores, which may range from 0 to 145, with a higher score signifying healthier [26]. Based on the total scale, the Cronbach's value was 0.91. The subscale coefficients ranged from 0.74 to 0.94. This study mainly focused on its vitality scale.

With a 0-3 rating scale, the HADS comprises 14 items and 2 dimensions (anxiety and depression). The total score for each dimension, calculated by summing the item scores, ranged from 0 to 21. Notably, no symptom is determined when the total score is less than 7 points, and the presence of symptoms is suspected or confirmed when equal to or more than 7 points. The values for the anxiety and depression dimensions of Cronbach's alpha were respectively 0.92 and 0.84.

PQSI comprises 18 self-rated items across 7 components. Each component was scored on a 3-point scale. By adding the component scores, the total score was obtained, which had a range of 0-21. Similarly, the points lower than 7 indicates normal sleep while those equal to or over 7 indicates a sleep disorder. The worse the sleep quality, the higher the score. As for the values of Cronbach's alpha, test-retest reliability and split-half reliability coefficient of the overall scale were 0.85, 0.99, and 0.82, respectively.

PSSS includes 12 items and 2 dimensions (intrafamilial and extrafamilial supports), scored on a 7-point scale, which ranged from 1 (indicating no) to 7 (indicating strongly agree). Total scores, calculated by adding the item scores, ranged from 7 to 84. Better perceived social support was indicated by a higher score. In terms of Cronbach's alpha, the total, intrafamilial, and extrafamilial support scales respectively had values of 0.92, 0.85, and 0.91.

Behavioral self-management has 25 items scored on a four-point rating scale. The overall scale includes ten dimensions: compliance with recommendations for sodium, protein, iron, and liquid intake; self-monitoring disease; forming good habits; protecting the internal fistula; maintaining personal health; seeking knowledge; developing interests and hobbies; and compliance with medication regimens. Calculated by adding the item scores, total scores had a range of 25-100. Noticeably, the behavioral self-management was better when the score was higher. By the way, the test-retest reliability was 0.93, and the value of Cronbach's alpha was 0.80.

### 2.5. Sample Size and Power

The sample size was based on a comparison of the mean between two samples (*N* = [2 (*U*_*α*/2_ + *U*_*β*_) *σ*/*δ*]^2^). The primary outcome was fatigue, assessed by the RPFS. According to related studies in the literature [27, 28], the numerical range of *δ* was estimated to be between 1.1 and 2.2, indicating a significant difference, and the numerical range of *σ*2 was estimated to be between 2.1 and 3.4. Assuming a two-tailed test with *α* of 0.05 and power of 0.8, a necessary total sample size of 80 to 120 was calculated. Considering the circumstances of real-time patients in the dialysis center, we chose the midpoint value of 100 samples as the minimum sample size, allowing for an attrition rate of 20%. Overall, we exceeded this requirement by recruiting 120 participants.

### 2.6. Data Analysis

Under the guidance of a statistician using the SPSS version 20.0 software, all statistical analyses were conducted. Mean ± standard deviation (SD) was used to describe the continuous variables displaying a normal distribution and the median and interquartile range to describe those displaying a skewed distribution. Differences in continuous variables with a normal distribution between groups were compared using independent-sample *t*-tests or those with a nonnormal distribution using Mann-Whitney *U* tests. A two-tailed *P* value < 0.05 was deemed as the threshold for statistical significance.

## 3. Results

### 3.1. Description of Studies

As shown in Figure 1, 168 patients were screened at our hospital's dialysis center. Of them, 48 patients were not interested in participating in this research. Thus, 120 hemodialysis recipients with fatigue who met the inclusion criteria and agreed to participate were randomized, with 64 patients in the experimental group and 56 in the control group. Two patients per group dropped out during the study. Ultimately, 116 participants were analyzed.

### 3.2. Sociodemographic and Individual Characteristics of Patients

The average age of the patients shown in Table 1 in this study was 56.39 ± 15.95 years, 56.03% were male, and 43.97% were female. The prevalence of fatigue was 61.29% and 62.96% in the experimental and control groups, respectively; 42 (36.21%) members of the experimental group and 30 (25.87%) members of the routine care group were <60 years old. The other baseline parameters of the participants are summarized in Table 1. Overall, the parameters were well balanced between the two groups.

As shown in Table 2, both groups had moderate total fatigue scores (5.71 *vs.* 5.79), and their mental fatigue was more severe than their physical fatigue (6.23 *vs.* 5.12 and 6.31 *vs.* 5.26, respectively). The level of behavioral self-management (61.07 *vs*. 60.50) was moderate or higher, and the level of vitality (13.03 *vs.* 13.43) was moderate. Simultaneously, clinical indicators such as the levels of serum hemoglobin (101.83 *vs.* 103.90), albumin (38.43 *vs.* 38.25), and calcium (2.07 *vs.* 2.07) were lower than normal in hemodialysis recipients with fatigue. The other symptoms, characteristics, and clinical indicators of the participants are summarized in Table 2.

### 3.3. Nurse-Led Nonpharmacological Integrative Interventions plus Standard Care Were More Beneficial Than Standard Care Only

There were significant differences after 6-month intervention in overall fatigue, mental fatigue, physical fatigue, vitality, sleep disorders, depression, overall behavioral self-management, compliance with sodium, protein, liquid, and iron intake recommendations, TSAT, and urea between the two groups (*P* < 0.05). Among these, the experimental group had much greater change in overall fatigue than the control group (*P* ≤ 0.001), and the between-group comparison of appetite after the 6-month intervention also presented a significant difference (*P* < 0.05) (Table 3).

## 4. Discussion

In the current study, we performed a parallel randomized controlled trial to explore the effects of a nurse-led nonpharmacological hybrid intervention for hemodialysis patients with fatigue. We found that the nonpharmacological integrative intervention significantly improved dietary compliance, medication adherence, and self-management skills to alleviate overall fatigue, enhance self-management behavior, and improve various clinical biochemical indicators. These results indicated that each method of integrated care protocol influenced and promoted each other, which was in agreement with the combined interventions of aerobic exercise and acupoint massages, and was significantly more effective than aerobic exercise alone in alleviating cancer-related fatigue and normalizing serum phosphate levels [29]. Altogether, with advances in technology, implementing the nurse-led nonpharmacological intervention with standard care might have promising prospects in helping patient recovery and care, as well as reducing psychological burdens, including fatigue.

In 2015, the Kidney Disease Outcomes Quality Initiative guidelines reported that the assessment and supportive care management of symptoms of kidney disease should include the routine care of chronic kidney disease and that exercise training should be part of the comprehensive management of symptoms in patients treated with hemodialysis. Exercise interventions might be more effective than routine care in mitigating fatigue among hemodialysis adults, as reported by a systematic review [30]. Meanwhile, related research demonstrated that the prospect of energetic activity might be a demotivating factor for patients from continuing exercise training; a less vigorous exercise regimen was more appropriate for hemodialysis patients with fatigue [18]. In addition, the American Academy of Sports Medicine guidelines state that home walking training is a low-cost, easy, and convenient form of physical activity. Moreover, walking is considered a form of mild-intensity exercise training, which may improve not only physical functional status but also improve mental functional status [18]. Its possible mechanism might be that walking could improve cardiac function, accelerate the transport of various solutes by enhancing the perfusion of tissues across various organ systems, and thus speed the entry of large metabolites into the bloodstream for elimination, finally enhancing the ability of dialysis to ameliorate overall fatigue and other symptoms [31, 32], indirectly leading to the results that before and after the 6-month intervention the intervention group showed higher difference values of transferrin saturation and urea than the control group, along with other obvious differences found between the two groups.

Self-management, that is, daily health-related care performed by patients with chronic diseases, is critical to effective care of chronic diseases [33]. Self-efficacy is an essential component of self-management [34], and increasing self-efficacy had a meaningful effect on the improvement of patients' self-care behavior [35], thereby enhancing their capacity to participate in healthy behaviors and follow treatment recommendations [34]. Accordingly, a meta-analysis showed that improving the self-management of fluid intake and diet restrictions in hemodialysis patients exerted indirect control over interdialytic weight gain, thus reducing fatigue [36].

Moreover, self-efficacy in self-management was shown to predict the improvement of health behavior, which was positively associated with medication adherence, dialysis adherence, and self-care behaviors, enabling patients to gain the full benefit of dialysis and promoting the elimination of metabolites to ameliorate overall fatigue and other symptoms [31, 32]. Bonner et al. [37] verified that self-management programs might improve the health-related quality of life of patients on hemodialysis. Similar changes were observed in our study, with the intervention enhancing self-management behavior and reducing overall fatigue and some other indicators in patients with fatigue on hemodialysis. Therefore, the behavioral self-management education in our research was intended to help hemodialysis patients relieve fatigue, indirectly reduce the cost of the disease, and enhance longevity and quality of life by increasing the self-care skills of hemodialysis patients [36].

In addition, MI, a psychological intervention that can be delivered by personnel without specialized psychological qualifications, is a key component of long-term disease management [38]. The principle of MI is to help patients overcome ambivalence that stops them from changing their beliefs to adopt behavioral changes, such as improving adherence to dietary recommendations, to reduce disease complications and enhance the quality of life [39]. Therefore, MI, as part of the holistic care intervention in this study, would first promote cognitive changes in hemodialysis patients with fatigue and then lead to behavior changes such as sustaining a walking regimen and adhering to self-management protocols, ultimately resulting in perceived bodily wellness as reflected by reductions in fatigue and other symptoms. This was in agreement with the results of meta-analyses and systematic reviews showing that physical activity, adherence, communication, and other numerous symptoms were effectively improved by MI-based interventions [40, 41]. Additionally, a prior study stated that self-efficacy in self-management was positively linked to patient initiative in making lifestyle changes to achieve goals [42], which was consistent with our study results.

The present study had some limitations. After the end of the intervention, there was no long-term follow-up. The intervention group may have received much more staff attention than the control group. The current investigation was only a single-center study with limited sample size. The intervention process and results had no quality control for the effects of having a nurse intervention. Therefore, we will need to conduct multicenter studies and long-term follow-ups to verify the effects of nonpharmacological nurse-led integrated care protocols. Meanwhile, we recommend future research to dig out the biological mechanism of fatigue in patients undergoing hemodialysis and test whether specific biochemical indicators are involved in the benefit of nonpharmacological nurse-led integrated care protocols for hemodialysis patients with fatigue.

## 5. Conclusions

The results suggested that the nonpharmacological holistic care intervention used in this study, involving a well-rounded multidisciplinary team, can improve dietary compliance, medication adherence, and self-management skills to alleviate overall fatigue, enhance self-management behavior, and improve various clinical biochemical indicators. Meanwhile, the dialysis nurses were permeated through interventions, and the role and function of nurse-led intervention were also displayed in this study.

## Figures and Tables

**Figure 1:** CONSORT flow diagram of the study. Abbreviation: MI: motivational interviewing.

**Table 1:** Baseline characteristics of the two groups before intervention (categorical data, *n* = 116).

Variable	Type	Overall sample	Intervention group (*n* = 62)	Control group (*n* = 54)	*P* value
Fatigue		72 (62.07)	38 (61.29)	34 (62.96)	0.853

Gender	Male	65 (56.03)	31 (50.00)	34 (62.96)	0.161

Age (years)	<60	72 (62.07)	42 (67.74)	30 (55.56)	0.177

Ethnicity	Han	44 (37.93)	24 (38.71)	20 (37.04)	0.853

Comorbidities	≥3	46 (39.66)	24 (38.71)	22 (40.74)	0.832

Living situation					0.326
	Alone	14 (12.07)	6 (9.68)	8 (14.81)	
	Husband and wife	39 (33.62)	26 (41.94)	13 (24.07)	
	With parents	11 (9.48)	7 (11.29)	4 (7.41)	
	With children	44 (37.93)	19 (30.65)	25 (46.30)	
	With siblings	2 (1.72)	1 (1.61)	1 (1.85)	
	With parents and children	6 (5.17)	3 (4.84)	3 (5.56)	

Marital status					
	Unmarried	6 (5.17)	3 (4.84)	3 (5.56)	
	Married	93 (80.17)	48 (77.42)	45 (83.33)	
	Divorced	4 (3.45)	2 (3.23)	2 (3.70)	
	Separated	5 (4.31)	3 (4.84)	2 (3.70)	
	Widowed	8 (6.90)	6 (9.68)	2 (3.70)	

Employment	Yes	4 (3.45)	2 (3.23)	2 (3.70)	1.000

Education					0.977
	Below elementary school	14 (12.07)	4 (6.45)	10 (18.52)	
	Elementary school	31 (26.72)	16 (25.81)	15 (27.78)	
	Middle school	35 (30.17)	20 (32.26)	15 (27.78)	
	High school or secondary school	14 (12.07)	6 (9.68)	8 (14.81)	
	Junior college, undergraduate, or above	22 (18.97)	16 (25.81)	6 (11.11)	

Family income (RMB/month)					0.489
	≤900	31 (26.72)	15 (24.19)	16 (29.63)	
	901-1500	20 (17.24)	12 (19.35)	8 (14.81)	
	1501-3000	22 (18.97)	15 (24.19)	7 (12.96)	
	3001-5000	24 (20.69)	11 (17.74)	13 (24.07)	
	≥5001	19 (16.38)	9 (14.52)	10 (18.52)	

Means of paying medical expenses					0.184
	Own expense	4 (3.45)	2 (3.23)	2 (3.70)	
	Medical insurance	51 (43.97)	30 (48.39)	21 (38.89)	
	Free medical service	7 (6.03)	6 (9.68)	1 (1.85)	
	Rural cooperative medical service	54 (46.55)	24 (38.71)	30 (55.56)	

Exercise	Yes	51 (43.97)	29 (46.77)	22 (40.74)	0.514

Exercise time					0.228
	<30 min	84 (72.41)	42 (67.74)	42 (77.78)	
	≥30 min	32 (27.59)	20 (32.26)	12 (22.22)	

Complications	Yes	97 (83.62)	54 (87.10)	43 (79.63)	0.278

Pain (whole body)	Yes	44 (37.93)	23 (37.10)	21 (38.89)	0.843

Pruritus	Yes	94 (81.03)	50 (80.65)	44 (81.48)	0.909

Appetite					0.594
	Poor	46 (39.66)	23 (37.10)	23 (42.59)	
	General	46 (39.66)	24 (38.71)	22 (40.74)	
	Normal	24 (20.69)	15 (24.19)	9 (16.67)	

Dialysis frequency (times/week)					0.072
	1 time/week	4 (3.45)	0	4 (7.41)	
	2 times/week	59 (50.86)	36 (58.06)	23 (42.59)	
	3 times/week	22 (18.97)	12 (19.35)	11 (20.37)	
	4 times/week	6 (5.17)	2 (3.23)	4 (7.41)	
	5 times/two weeks	25 (21.55)	12 (19.35)	12 (22.22)	

*Note*: data was expressed as *n* (%). Fisher's exact test and Pearson chi-square test.

**Table 2:** Comparison of preintervention baseline characteristics between groups (continuous data, *n* = 116).

Characteristic	Intervention group (*n* = 62)	Control group (*n* = 54)	Comparison (*P* value)
Overall fatigue^a&^	5.71 ± 1.51	5.79 ± 1.86	0.863
Muscular fatigue^&^	5.12 ± 1.55	5.26 ± 2.07	0.774
Mental fatigue^&^	6.23 ± 1.92	6.31 ± 1.97	0.881
Overall perceived social support^b&^	52.33 ± 13.58	53.96 ± 13.54	0.649
Extrafamilial support^&^	28.90 ± 12.17	31.14 ± 11.90	0.481
The vitality of SF-36^c&^	13.03 ± 4.42	13.43 ± 3.88	0.720
PQSI^d&^	12.20 ± 4.11	11.93 ± 3.64	0.791
Depression^e&^	9.57 ± 6.27	10.82 ± 4.83	0.399
Overall self-management behavior^f&^	61.07 ± 10.96	60.50 ± 10.20	0.462
Compliance with recommendations for liquid intake^&^	12.47 ± 4.21	12.57 ± 4.55	0.928
Hb (g/L)^&^	101.83 ± 21.98	103.9 ± 21.39	0.462
ALB (g/L)^&^	38.43 ± 3.66	38.25 ± 2.90	0.708
P (mmol/L)^&^	1.95 ± 0.49	2.07 ± 0.51	0.057
Ca (mmol/L)^&^	2.07 ± 0.25	2.07 ± 0.25	0.829
Fe (*μ*mol/L)^&^	10.23 ± 4.86	10.00 ± 5.35	0.705
TSAT^&^	29.37 ± 9.91	29.12 ± 8.58	0.845
	Median (*P*25, *P*75)	Median (*P*25, *P*75)	
CRP (mg/L)^#^	4.61 (0.44, 12.96)	2.67 (0.34, 11.43)	0.808
PTH (pg/mL)^#^	357.90 (159.2, 529.93)	391.90 (149.23, 652.73)	0.529
SF (*μ*g/L)^#^	219.90 (59.78, 504.50)	220.65 (54.58, 686.85)	0.919
Urea (mmol/L)^#^	9.72 (6.34, 20.88)	8.44 (5.99, 20.88)	0.231
Intrafamilial support^g#^	24.00 (20.00, 28.00)	24.00 (22.00, 24.00)	0.703
Anxiety^h#^	3.00 (1.75, 5.00)	2.50 (0.25, 4.75)	0.339
Compliance with recommendations for sodium and protein intake^#^	15.50 (11.75, 17.00)	17.00 (12.50, 17.00)	0.506
Compliance with recommendations for iron intake^#^	5.00 (3.00, 6.50)	3.00 (3.00, 5.00)	**0.042**
Self-monitoring disease^#^	6.00 (4.75, 6.25)	6.00 (5.25, 7.75)	0.515
Developing good habits^#^	5.00 (5.00, 6.25)	5.00 (5.00, 5.00)	0.139
Protecting internal fistula^#^	3.50 (1.00, 4.00)	4.00 (2.00, 4.00)	0.287
Maintaining personal health^#^	5.00 (4.00, 5.25)	4.00 (3.25, 4.00)	0.373
Seeking knowledge^#^	5.00 (2.00, 7.00)	5.00 (3.00, 7.00)	0.589
Developing interests and hobbies^#^	1.00 (1.00, 1.00)	1.00 (1.00, 1.00)	0.283
Compliance with medication regimen^#^	4.00 (4.00, 4.00)	4.00 (4.00, 4.00)	1

Abbreviations: Hb: hemoglobin; ALB: albumin; P: phosphorus; Ca: calcium; Fe: ferritin; SF: serum ferritin; TSAT: serum transferrin saturation; SF-36: 36-Item Short-Form Health Survey; PSQI: Pittsburgh Sleep Quality Index; CRP: C-reactive protein; PTH: parathyroid hormone; SF: serum ferritin; Ur: urea. Bold values are statistically significant (*P* < 0.05). ^a^Total scores can range from 0 to 10, of which 0, 1–3, 4–6, and 7–10 indicate no symptoms, mild symptoms, moderate symptoms, and severe symptoms, respectively. ^b^Total support scores can range from 12 to 84, with higher scores indicating better perceived social support. ^c^Total scores can range from 0 to 145, with higher scores indicating better health. ^d^Total scores can range from 0 to 21, with ≤7 points indicating normal sleep and >7 points indicating a sleep disorder. ^e^Total scores can range from 0 to 21, with <7 points indicating no symptoms and ≥7 points indicating that symptoms are suspected or confirmed. ^f^Total scores can range from 25 to 100, with a higher score indicating better behavioral self-management. ^g^Intrafamilial support scores ranged from 4 to 28, with higher scores indicating better perceived social support. ^h^Total scores can range from 0 to 21, with <7 points indicating no symptoms and ≥7 points indicating that symptoms are suspected or confirmed. ^&^The variables were normally distributed and are expressed as the mean ± standard deviation (SD). Two-tailed independent-sample *t*-test, *P* > 0.05. ^#^The variables were nonnormally distributed and are displayed as the median ± IQR, where the IQR is the difference between the 25th percentile (*P*25) and the 75th percentile (*P*75). Mann-Whitney *U* test, *P* > 0.05.

**Table 3:** Comparison of the difference values between the two groups pre- and postintervention (*n* = 116).

Indicators	Median (*P*25, *P*75)	Median (*P*25, *P*75)	Comparison (*P* value)
	Intervention group (*n* = 62)	Control group (*n* = 54)	
Overall fatigue^ag^	2.25 (1.43, 3.43)	0.50 (0.27, 1.05)	≤0.001
Mental fatigue^g^	1.31 (0.51, 2.89)	0.64 (0.22, 1.12)	≤0.001
Muscular fatigue^g^	2.06 (1.25, 3.00)	0.79 (0.24, 1.18)	≤0.001
CRP (mg/L)	1.84 (-2.22, 8.30)	1.31 (-3.41, 4.37)	0.213
PTH (pg/mL)	22.66 (-27.37, 64.01)	9.40 (-26.38, 67.50)	0.656
Hb (g/L)	8.00 (-2.00, 28.00)	5.50 (1.75, 23.00)	0.737
ALB (g/L)	6.17 (1.13, 8.34)	4.42 (1.72, 8.58)	0.646
P (mmol/L)	0.32 (-0.44, 1.01)	-0.05 (-0.33, 0.29)	0.185
Ca (mmol/L)	0.18 (-0.06, 0.47)	0.10 (-0.11, 0.30)	0.138
Fe (*μ*mol/L)	3.19 (-2.19, 7.64)	0.76 (-1.78, 4.66)	0.188
SF (*μ*g/L)	25.36 (-12.38, 52.66)	10.65 (-13.04, 29.16)	0.301
TSAT^g^	8.03 (2.25, 14.87)	2.06 (0.79, 2.89)	≤0.001
Urea (mmol/L)^h^	3.35 (-0.07, 11.73)	1.62 (-3.47, 5.97)	**0.018**
PSSS^b^	6.00 (2.75, 6.00)	5.00 (-16.00, 21.00)	0.876
Intrafamilial support	4.00 (2.00, 4.00)	2.00 (0.00, 6.00)	0.359
Extrafamilial support	2.00 (-16.00, 16.00)	2.00 (0.00, 2.00)	0.965
Vitality on the SF-36^h^	5.00 (1.00, 9.00)	2.00 (2.00, 5.25)	**0.048**
PQSI^ch^	4.00 (0.75, 6.00)	1.00 (0.00, 3.00)	**0.002**
Anxiety	1.00 (-2.00, 4.00)	1.00 (0.00, 1.00)	0.616
Depression^h^	2.50 (0.00, 6.25)	1.00 (0.00, 3.00)	**0.012**
Overall behavioral self-management^dg^	16.50 (6.00, 19.25)	6.50 (2.00, 12.00)	≤0.001
Compliance with recommendations for sodium and protein intake^h^	3.00 (1.00, 5.00)	1.00 (0.00, 4.00)	**0.001**
Compliance with recommendations for liquid intake^h^	3.00 (1.00, 7.00)	2.00 (0.00, 3.25)	**0.005**
Compliance with recommendations for iron intake^g^	2.00 (0.00, 3.00)	0.00 (0.00, 0.00)	≤0.001
Self-monitoring of disease	1.00 (0.00, 3.00)	0.00 (0.00, 1.00)	0.146
Developing good habits	0.00 (0.00, 1.00)	0.00 (0.00, 1.00)	0.337
Protecting the internal fistula	0.00 (0.00, 1.00)	0.00 (0.00, 1.00)	0.399
Maintaining personal health	1.00 (0.00, 2.00)	0.00 (0.00, 1.00)	0.064
Seeking knowledge	0.00 (-2.00, 3.00)	0.00 (0.00, 1.00)	0.877
Developing interests and hobbies	0.00 (0.00, 1.00)	0.00 (0.00, 0.00)	0.424
Compliance with medication regimen	0.00 (0.00, 0.00)	0.00 (0.00, 0.00)	1

Abbreviations: CRP: C-reactive protein; PTH: parathyroid hormone; Hb: hemoglobin; ALB: albumin; P: phosphorus; Ca: calcium; Fe: ferritin; SF: serum ferritin; TSAT: serum transferrin saturation; SF-36: 36-Item Short-Form Health Survey; PSSS: Perceived Social Support Scale; PSQI: Pittsburgh Sleep Quality Index. The continuous within-group variables are reported as the median ± interquartile range of difference values between pre- and postintervention measurements; the categorical variables are expressed as frequencies after the intervention. Bold values are statistically significant (*P* < 0.05 or *P* < 0.01). ^a^Total fatigue scores can range from 0 to 10, of which 0, 1–3, 4–6, and 7–10 indicate no symptoms, mild symptoms, moderate symptoms, and severe symptoms, respectively. ^b^Total support scores can range from 12 to 84, with higher scores indicating better perceived social support. ^c^Total scores can range from 0 to 21, with ≤7 points indicating normal sleep and >7 points indicating a sleep disorder. ^d^Total scores can range from 25 to 100, with a higher score indicating better behavioral self-management. ^g^Comparison of the difference values of pre- and postintervention between groups, *P* < 0.001. ^h^Comparison of the difference values of pre- and postintervention between groups, *P* < 0.05.

## Data Availability

The raw datasets analyzed in this study are available from the corresponding author on reasonable request after deidentification.
